# SARS-CoV-2 Transmission by Arthropod Vectors: A Scoping Review

**DOI:** 10.1155/2022/4329423

**Published:** 2022-08-08

**Authors:** Shahin Nekoei, Faham Khamesipour, Marlene Benchimol, Rubén Bueno-Marí, Davood Ommi

**Affiliations:** ^1^Faculty of Veterinary Medicine, Shahrekord Branch, Islamic Azad University, Shahrekord, Iran; ^2^Center for Research and Training in Skin Diseases and Leprosy, Tehran University of Medical Sciences, Tehran, Iran; ^3^Universidade do Grande Rio (Unigranrio), Rio de Janeiro, Duquxe de Caxias, Rio de Janeiro, Brazil; ^4^Department of Research & Development (R&D), Laboratorios Lokímica, Valencia, Spain; ^5^Parasitology Area, Department of Pharmacy and Pharmaceutical Technology and Parasitology, University of Valencia, Burjassot (Valencia), Spain; ^6^Functional Neurosurgery Research Center, Shohada-e Tajrish Neurosurgical Center of Excellence, Shahid Beheshti University of Medical Sciences, Tehran, Iran

## Abstract

COVID-19 is a respiratory disease of worldwide importance as it has brought enormous health problems to the world's population. The best-known way of transmission of the virus is through aerosolization. However, research is needed to explore other transmission routes. Researchers hypothesized that arthropods could transmit SARs-CoV-2. This study is aimed at reviewing research on arthropods as possible reservoirs and/or vectors of SARS-CoV-2, the causative agent of COVID-19. Following PRISMA guidelines, we conducted a systematic review using several electronic databases/academic searches with the search terms “arthropods,” “coronavirus,” and “transmission.” A total of 64 unique articles were identified, of which 58 were included in the review. The SARS-CoV-2 virus is tiny and invisible to the naked eye, and its presence in stools, droplets, and surfaces was detected. One doubt is whether insects can transmit the virus from one place to another. Thus, a healthy carrier of the COVID-19 virus can be at the root of the contamination of their community or their family through the transport of the virus by insects from the interior (flies, cockroaches, etc.) from their feces and food surfaces. Hygiene care within communities and families becomes a prime factor. Coronavirus infection is a significant public health problem around the world. The prevention and control of outbreaks remain very important, even with the production of new vaccines. The main option to achieve this is the proper management of the transmission of the virus. The registry of infected people is currently the basis for the transmission of COVID-19. However, questions about the possibility of infection from other sources and its prevention are not receiving adequate attention. Numerous studies have shown the possibility that SARS-COV-2 fragments could have a longer life than shed respiratory droplets. Also, this virus is larger than those of other coronavirus families.

## 1. Introduction

COVID-19 is an emerging respiratory infection in humans, with the causative agent identified as SARS-CoV-2 [1]. The virus has substantially impacted public health and the global economy [2]. While the initial source of SARS-CoV-2 transmission to humans is still being debated, it is believed that this initial event (or events) was from animals to humans [3–5]. Human-to-human transmission is the major route of virus transmission to people [6]. To date, vertical transmission has not been confirmed, but several cases of postnatal transmission have been reported [7]. Worldwide, more than one billion zoonotic diseases occur yearly, putting pressure on global health systems, economies, and environmental resources [8, 9]. Thus, surveillance and prevention of these diseases are fundamental to reducing the impact of future epidemics [10]. The diversity of animal reservoirs is a challenge in controlling pathogen spread, with animal reservoirs allowing these agents to perpetuate more easily [9]. The incidence of emerging infectious diseases (EIDs) has increased over the past 20 years and may continue to grow. EIDs may be caused by known or newly identified pathogens and represent at least 12% of pathogens found in humans [9, 10].

Examples of SIAs include West Nile Fever, influenza, severe acute respiratory syndrome (SARS), and the Middle East Respiratory Syndrome coronavirus (MERS-CoV) [11]. Wildlife species can be reservoirs for pathogens that threaten public health [9, 11]. Consequently, human activities and lifestyles increase interactions between humans and wildlife, facilitating the spread of infectious agents to new hosts and habitats, establishing new and potentially dangerous relationships, and changing existing ecological niches in disease transmission cycles [9]. Environmental contamination has been proposed for transmitting SARS-COV-2 in healthcare professionals (HCWs) [12]. COVID-19 virus is related to the bat coronavirus. It was developed that the transmission and evolution of the COVID-19 virus were from bats to pangolins and then to humans [13]. The scientific investigation leads us to believe that COVID-19 is transmitted by respiratory droplets, aerosols, and human-to-human contact. In addition, there is a possibility of contamination by the oral-fecal route.

There are currently several vaccines available for COVID-19 infections. According to worldwide statistics, the disease's mortality rate is 3.4%. [1, 5, 14, 15]. Scientific experiments have shown that contaminated droplets can transmit SARS-COV-2 in the air. However, the participation of insects in transmission and environmental contamination is still not well elucidated [16]. It is important to note that close contact between patients and insects may occur in hospitals [17].

Arboviral diseases (viral diseases transmitted by arthropods) include many RNA viruses with a life cycle requiring both a host (bird or mammal) and an arthropod vector [18]. Arbovirus replication occurs in their vertebrate hosts and arthropods. Blood-sucking arthropods are responsible for transmission between vertebrates.

No studies have reported transmission of SARS-CoV-2 by blood-sucking arthropods such as mosquitoes [19–23]. However, contaminated individuals' feces or personal use materials may be promising sources of viral transmission through flies and cockroaches [24–26]. This review is aimed at presenting the available information on SARS-CoV-2 transmission by vectors.

## 2. Materials and Methods

### 2.1. Search Strategy

This review adheres to the Preferred Reporting Items for Systematic Reviews and Meta-Analyses extension for scoping reviews (PRISMA-ScR) reporting. The keywords “arthropods,” “Coronavirus,” and “transmission” were entered into PubMed, Scopus, Google Scholar, and MedLine. The search strategy was based on three components: (1) transmission route, (2) insects (arthropods) participating in the transmission or dispersal of etiological agents of human diseases (COVID-19), and (3) prevention, implication, and control. The search filters were developed based on suggestions from the thesaurus of the MeSH (Medical Subject Headings) term platform of the PubMed/Medline digital library (US National Library of Medicine National Institute of Health). Later, these descriptors were adapted to the Scopus and SciELO (Scientific Electronic Library Online) platforms. The following descriptors and Boolean operators were used: “wild animals AND COVID-19's transmission,” “zoonosis AND COVID-19,” and “COVID-19 AND wild animals.” There was no language or publication date restrictions. Duplicate articles have been eliminated. After the first selection, all potentially relevant scientific articles were downloaded to assess their eligibility.

### 2.2. Data Extraction, Exclusion, and Inclusion Criteria

Articles were excluded if the (1) studies discussed COVID-19 but had explained wild animals (insects or Arthropods) as transmission way, (2) COVID-19 transmission was related to insects, and (3) studies involve incomplete texts, review articles with no new data, editorials, master's or doctoral theses, and book chapters. In addition, the references to included articles were evaluated for other potentially relevant documents. The criteria for inclusion of articles were as follows: (1) must be an analysis of data on COVID-19 and (2) must encompass some relationship between the transmission of COVID-19 and insects.

The following information was recorded for the included studies: (1) publication characteristics—author, year, journal, and country; (2) animal characteristics—species; and main results of the study.

## 3. Results

A total of 78 articles were identified. After a first sort which made it possible to eliminate duplicate articles, we, therefore, retained 64 articles. An in-depth reading of the articles led to the second selection of 58 articles for this study.  Figure 1 shows the item selection diagram according to the PRISMA statement.

### 3.1. Economic Impact of COVID-19

Today, the global economy is hit by the worst recession due to the pandemic, which is seen as one of the world's greatest collective failures. The COVID-19 pandemic and society's responses are weakening economies worldwide, experiencing demand, and supply shocks. The most severe economic consequences in history since the Great Depression are expected. Growth forecasts for the Indian economy were revised downwards by the International Monetary Fund (IMF) in April 2020, thus projecting a GDP growth of 1.9% in 2020 [27–29]. COVID-19 has caused many people from all over the world to review their daily life habits.

In response to travel bans and various restrictive measures governments worldwide take to curb the spread of the virus, many people are adopting digital tools to maintain normality. According to the International Labor Organization, there could be a growth in employment worldwide (from 5.3 million to 24.7 million) due to the economic crisis and the work paralysis that resulted from the COVID-19 pandemic. The global impact is expected to be between $77 and $347 billion or 0.1 to 0.4 percent of global GDP [30].

### 3.2. Transmission of SARS-CoV-2

The coronavirus is an animal virus endowed with an envelope with a positive-sense single-stranded RNA and a genome size of 26 to 32 kb; they belong to Coronaviridae, order Nidovirales, and genus Betacoronavirus [14]. Human Coronavirus 229E (HCoV-229E), NL63 (HCoV-NL63), OC43 (HCoV-OC43), HKU1, MERS-CoV, SARS-CoV, and the most recent SARS-CoV-2 or CoV-2019 or COVID-19 virus or novel corona-2019 virus are the seven types of human coronaviruses commonly identified among infected people worldwide and cause respiratory infections in the population (children and adults) [19, 31]. COVID-19 is related to a bat coronavirus. Scientifically, it has been reported that COVID-19 has been transmitted from bats to pangolins and then to humans [32]. Infection with respiratory viruses can occur through contact, droplet spray, and aerosol [33] (Table 1). Transmission can also occur through coughing, sneezing, and hand contact with patients' faces (nose, eyes, and mouth). Transmission can also occur through contact with the surface of objects or equipment belonging to patients or contaminated. [13]. Data analysis suggests that closer contact between individuals is necessary to facilitate the spread of SARS-CoV-2 [18].

According to the United States Centers for Disease Control and Prevention, COVID-19 is a new disease, and we do not yet fully understand how it is spread [20]. Our current and primary understanding is that the virus spreads primarily between people via respiratory droplets from the coughing and sneezing of an infected person from about six feet away. Despite this, some experts believe that a height of 1.8 meters (6 feet) is still insufficient [34]. Air currents affect the movement of respiratory droplets. Larger droplets over 5 *μ*m do not remain in the air for long periods and move over small distances, typically less than 1 m (less than 3.3 feet) [35–37]. Small droplets (<5 *μ*m) can remain suspended in the air for a long time and travel significant distances, going beyond 1 m (more than 3.3 feet) [38].

In addition to transmission of COVID-19 through respiratory droplets, close contact, and aerosols, scientists are also raising possible fecal-oral transmission. Furthermore, patients may pass the virus to others during incubation [39]. But there have been no reports of transmission of COVID-19 by hematophagous arthropods such as mosquitoes [23]; since then, Dutto et al. described the importance of insects in the transmission of COVID-19. So what are the possible mechanisms of transmission of the COVID-19 virus by arthropod insects?

### 3.3. Arthropod Vectors of Transmission of the COVID-19 Virus: What Mechanisms?

Insects, crustaceans, arachnids, and myriapods constitute the classes of arthropods [40].

In nature, insects are abundant, which can be harmless or live as parasites. Parasitic arthropods are often vectors for disease transmission, as they feed primarily on the blood of animals and humans [41]. However, there is no evidence that an arthropod that has taken its blood meal from a diseased host is not infected, nor that the pathogens it has potentially ingested can survive and grow.

Coronavirus disease originated in animals before it was transmitted to humans. Transmission of these viruses can occur through direct contact with an infected animal or through the consumption of food or other products that do not receive adequate care. In any case, there is no evidence of this type of transmission by insects.

Thus, until there is evidence to the contrary, insects may be potential virus vectors, and we should be wary of them [41]. Most indoor insects are potential vectors and can play a key role in transmitting infectious diseases. For example, tick bugs are very dangerous, as they are often vectors of encephalitis, which killed over 150,000 people in 2015 alone. The tick can infect any animal or human during its life. Both can then infect other individuals in a noninvasive way [18]. Flies contaminate food and infect animals and humans through the skin. More than 60 diseases worldwide are linked to flies. The infective role of flies is well known, which can act as transmitters of diseases both for food and for parts of the body such as open wounds, eyes, nose, and mouth [42]. Fleas were the vectors mainly incriminated in the spread of the plague from antiquity to the Middle Ages. They are very mobile, can travel far, and can enter any place. They can transmit many pathogens to domestic animals and humans. These can include helminthiasis, encephalitis, and many others. Of course, the Middle Ages are history, but there is no evidence that fleas feeding on bats are not carriers of COVID-19 [18].

Cockroaches are among the most dangerous insects. They are nasty and agile insects; they reproduce very quickly and eat the rubbish that gets in their way. Belonging to the most notorious local pests, they can contaminate food by leaving droppings and bacteria that cause food poisoning. They also transmit bacteria, viruses, fungi, and other pathogenic microorganisms to infested areas [34]. In famous vectors of encephalitis, malaria, and several other dangerous and difficult to treat diseases, mosquitoes infect more than 200 million people in Asia, the Middle East, South America, and Africa. In addition, they can carry infected blood in their wombs and then infect many people [18].

No studies have been conducted on the transmission of COVID-19 by hematophagous arthropods such as mosquitoes and lice [21]. However, the role of flies and cockroaches in the mechanical transmission of microorganisms in contact with contaminated surfaces or even with the feces of sick people is well known. A few cases of the presence of the virus in the stools of patients have been reported [35, 36, 43]. SARS-CoV-2 has been detected at 53.4% in the stools of patients with COVID-19 [37, 38, 44]. In addition, despite the positivity of stool samples, 23% of patients were negative for the virus in respiratory samples [45]. Ninety-eight patients with COVID-19 exhibited viral shedding in the stool for nearly five weeks after negative respiratory samples [5]. Likewise, an elevation of SARS-CoV-2 in the stool can be observed in healthy carriers [38]. In a scientific investigation of cockroach-borne coronavirus, 15 cockroach surface swabs were tested, and a single uncertain positive result was obtained from nested RT-PCR [46]. Since feces can be a potential source of transmission of COVID-19, any organism that comes in contact with or feeds on human feces is likely to transmit COVID-19 even after it has tested negative because the virus is long-lived in the environment. Therefore, the involvement of insects in the transmission of COVID-19 must be considered [13].

### 3.4. Prevention and Control

SARS, MERS, and now SARS-COV-2 are zoonotic coronaviruses that can pass from animals to humans through direct contact with an infected host and indirect contact or consumption of contaminated food. Very common, zoonotic diseases can be spread by person-to-person contact once they have passed from animals to humans, making hand washing and other preventive actions outlined by the CDC imperative for public safety [47]. The possible virus transmission by insects in contact with patients and health workers is not mentioned in the WHO protocols for COVID-19. Several Chinese provinces have reported COVID-19 contamination in hospitals, prisons, and other crowded places [43]. Contamination of the environment, proximity, and contact of people in such places are important factors that can improve transmission [43, 48]. Controlling SARS-COV-2 and preventing its rampant spread is a global challenge that requires universal management. The management will go through personal, biological, and physical hygiene and less risk of chemical control. Therefore, it is important to ensure good environmental hygiene, especially the bathrooms, toilets, and kitchens preferential places for cockroaches and houseflies [49].

Eliminating cockroaches, flies, and mechanical vectors is important in every place, public or private. Environmental rehabilitation is in a good position among the procedures for controlling these vectors. Protecting surfaces with stainless steel or plastic screens, covering food containers, and using poison baits, light traps, and sticky traps are techniques for physical and mechanical control of these insects. Likewise, the effectiveness of medicinal plants such as *Veratrum nigrum* and *Eucalyptus* in repelling house flies, mosquitoes, and cockroaches is also demonstrated [36, 50, 51]. Garbage dumps, animal remains, garbage cans, etc. can serve as nests for houseflies and roaches to breed. To limit possible contact between insects and respiratory droplets, isolation and care centers should use mosquito nets to protect them.

### 3.5. Risk of SARS-CoV-2 Infection from Contaminated Water Systems

Could water contamination used in crops be contaminated with SARS-CoV-2 viral particles? SARS-CoV-2 viral RNA has been detected in infected persons' feces, and studies have also reported its occurrence in wastewater and surface water bodies [37, 52]. Therefore, water may be a possible route to virus outbreaks. It is important to mention that adequate water quality within irrigation practices is fundamental to preventing harm to plants and soils, maintaining food safety, and protecting public health, since agricultural irrigation is the largest water use globally. Therefore, it is crucial to analyze whether contamination, persistence, and dissemination of viral particles occur, especially in water used in irrigation, which could eventually contain fecal residues and thus contain SARS-CoV-2 particles. Research efforts concentrated on SARS-CoV-2 indicate that the risk of virus transmission from the aquatic environment may be nonexistent. However, a few studies have reported the presence of SARS-CoV RNA in soils. However, there are still no studies on detecting SARS-CoV-2 in crops. Various coronaviruses have been found in both treated and untreated water. Still, the survival and sustainability of SARS-CoV-2 in aqueous environments depend on many factors, such as initial viral load, type of medium, exposure to sunlight, temperature, and organic matter. It has been noted that some coronaviruses can be active and infectious in sewage and water for several weeks. The few studies reported show that SARS-CoV-2 RNA is present in raw wastewater (WW) and treated WW, mainly when disinfection is inefficient or absent [53].

## 4. Discussion

The coronavirus was observed in animals before its transmission to humans for the first time. This transmission can occur through direct contact with an infected animal or by consuming contaminated meat or other products. The COVID-19 virus can be spread through contact with large aerosol droplets, unprotected coughing, sneezing, hand contact with the nose, eyes, or mouth of patients, and objects and surfaces and patient-owned materials [43]. Previous studies have reported the survival of coronaviruses, including SARS, on environmental surfaces and objects [13].

Most indoor insects are potential vectors and may be involved in spreading infectious diseases [18]. For example, cockroaches and flies can infect an individual through another infected individual's contaminated surfaces and feces [25, 26]. Thus, the lack of hygiene in hospitals (poor biocleaning of patient rooms and surfaces, nonsterilization of medical equipment, and noncompliance with hand washing) can contaminate health workers and hospital users (healthy people). However, there is no evidence that they may or may not carry the virus. Nevertheless, it implies that insects potentially carry viruses and that we should be wary of them until scientific evidence is provided [54]. Therefore, decision-makers must improve or institute a more rigorous hospital hygiene policy within public and private health facilities.

A lot of explanation is still lacking on this transmission route, but it should be noted that stool is a potential source of transmission of COVID-19. Thus, any organism that comes into contact with the stool is a potential vector in the transmission of COVID-19. Therefore, the important role that insects could play in the transmission of COVID-19 should not be overlooked [18]. The food of house flies and cockroaches consists of human remains, ranging from food, droppings, vomit, and water droplets. Once in contact, these insects can transport these remains to an immediate or nearby environment [13]. Since the SARS-CoV-2 virus is tiny, invisible to the naked eye, its presence in stools, droplets, and surfaces, it is quite possible that these insects (flies, cockroaches) can transmit the virus from one place to another. Thus, a healthy carrier of the COVID-19 virus can be at the base of the contamination of his community or his family through the transport of the virus by insects of the interior (flies, cockroaches, etc.) from its excrements towards food and surfaces. Therefore, it justifies respecting hygiene rules even within communities and households.

The absence of studies on the mechanism of transmission of the COVID-19 virus involving arthropods (insects) and the unavailability or insufficiency of scientific information on the subject constituted a major limitation for this study. SARS-CoV-2 RNA in water environments might represent a risk of irrigation water contamination. Therefore, it is necessary to investigate the eventual persistence of SARS-CoV-2 in crops.

## 5. Conclusion

Coronavirus infection is a significant public health problem around the world. Despite discovering several vaccines, prevention, and control of outbreaks remain very important. And the main option to achieve this is the proper management of the transmission of the virus. Most scientific information on the transmission of COVID-19 is based on infected registered individuals. However, sufficient efforts are not being made to prevent and control possible transmission from other sources. Numerous studies have shown the viability of SARS-CoV-2 in human fragments of a longer life span than in respiratory droplets. It should also be considered that the virus is larger than those of other coronavirus families.

## Figures and Tables

**Figure 1:** PRISMA model study design process.

**Table 1:** Major accepted respiratory routes of transmission [17].

Transmission route	Elements involved and element characteristics	Characteristics/definition of transmission	References
Contact	Contaminated hands	Self-inoculation of mucous membranes by contaminated hands	[55]
Direct	Deposited on persons.	Virus transfer from one infected person to another	[56]
Indirect	Deposited on objects	Virus transfer through contaminated intermediate objects (fomites)	[43]
Airborne droplets	Droplets (>5 *μ*m)	Short-range transmission	[33]
	Remain only shortly in the air (<17 min)	Inoculation directe d'une personne naïve par toux/éternuements/respiration d'une personne infectée	
	Dispersed over short distances (<1 m)	Deposition mainly on mucous membranes and the upper respiratory tract	
Aerosol droplets	Aerosols, droplet nuclei (>5 *μ*m)	Long-range transmission (LRT)	[48]
	Remain in the air for an almost infinite amount of time	Inhalation of aerosols in a repairable size range	
	Dispersed over long distances (>1 m)	Deposition along the respiratory tract, including the lower airways	

## Data Availability

The data that support the findings of this study are available from the corresponding author, upon reasonable request.

## Abbreviations

EIDs: Emerging infectious diseases
SARS: Severe acute respiratory syndrome
MERS-CoV: Middle East Respiratory Syndrome Coronavirus
HCWs: Healthcare workers
MeSH: Medical Subject Headings
SciELO: Scientific Electronic Library Online
IMF: International Monetary Fund
HCoV-229E: Human Coronavirus 229E.
